# Preventative and Therapeutic Probiotic Use in Allergic Skin Conditions: Experimental and Clinical Findings

This article has been retracted.

**DOI:** 10.1155/2013/932391

**Published:** 2013-09-01

**Authors:** Öner Özdemir, Azize Yasemin Göksu Erol

**Affiliations:** ^1^Department of Pediatrics, Division of Allergy and Immunology, Research and Training Hospital of Sakarya University, Faculty of Medicine, Sakarya University, Adnan Menderes Caddesi, Sağlık Sokak No. 195, Adapazarı, 54100 Sakarya, Turkey; ^2^Department of Histology and Embryology, Faculty of Medicine, Afyon Kocatepe University, 03200 Afyonkarahisar, Turkey

## Abstract

Probiotics are ingested live microbes that can modify intestinal microbial populations in a way that benefits the host. The interest in probiotic preventative/therapeutic potential in allergic diseases stemmed from the fact that probiotics have been shown to improve intestinal dysbiosis and permeability and to reduce inflammatory cytokines in human and murine experimental models. Enhanced presence of probiotic bacteria in the intestinal microbiota is found to correlate with protection against allergy. Therefore, many studies have been recently designed to examine the efficacy of probiotics, but the literature on the allergic skin disorders is still very scarce. Here, our objective is to summarize and evaluate the available knowledge from randomized or nonrandomized controlled trials of probiotic use in allergic skin conditions. Clinical improvement especially in IgE-sensitized eczema and experimental models such as atopic dermatitis-like lesions (trinitrochlorobenzene and picryl chloride sensitizations) and allergic contact dermatitis (dinitrofluorobenzene sensitization) has been reported. Although there is a very promising evidence to recommend the addition of probiotics into foods, probiotics do not have a proven role in the prevention or the therapy of allergic skin disorders. Thus, being aware of possible measures, such as probiotics use, to prevent/heal atopic diseases is essential for the practicing allergy specialist.

## 1. Background

The interest in probiotic preventative/therapeutic potential in allergic disorders stemmed from the fact that probiotics have been shown to improve intestinal dysbiosis and permeability and to reduce inflammatory cytokines. Such effects would be desirable in treating allergic disorders including atopic dermatitis (AD). Therefore, several studies have been recently designed to examine the efficacy of probiotics in many allergic conditions, such as eczema and food allergies [1, 2]. Especially, the literature on the clinical probiotic use in other skin allergy reactions of human is very scarce. Therefore, this paper will mostly have to discuss the literature on the preventative and/or prophylactic role of probiotic use in AD.

### 1.1. Clinical and Experimental Essentials of Preventative and Therapeutic Probiotic Use in Allergic Skin Conditions

Including the first publication in 1997, over 40 randomized, double-blind, and placebo-controlled clinical trials were conducted to study the effects of various probiotics on treatment and prevention of allergic diseases. In total, more than 3000 individuals (including those in placebo groups) have participated in these studies so far. In the first-time study done by Majamaa and Isolauri in 1997, the administration of Lactobacillus (Lctbs) rhamnosus GG (LGG) to highly selected patients (age < 2 years, challenge-proven cow's milk allergy, and mild-to-moderate eczema) significantly improved the total scoring of AD severity index (SCORAD) score [3]. Later, the Finnish study of Kalliomäki et al. was the first report to describe that the frequency of AD in neonates treated with LGG was half that of the placebo [4]. However, these results have been lately questioned by other trials, which reported no difference in the development and therapy of AD in neonates supplemented with LGG or other probiotics. Therefore, an allergy preventative or therapeutic effect of probiotics in AD and allergic skin conditions could not be consistently established. The aim of this paper is to characterize current knowledge of probiotic use in skin allergy reactions, including their preventative/therapeutic role in AD.

As briefly mentioned above, there are good (animal) experimental and (human) clinical theoretical bases for using probiotics in the prevention and therapy of allergic skin conditions such as AD [5]. Germ-free animal models demonstrate that bacterial gut colonization is essential for maturation of immune function and induction of oral tolerance [6]. It has been proposed that a similar but a more subtle process may be occurring in human beings with progressively cleaner environments. Probiotic intestinal flora is arguably the most abundant source of early immune stimulation and contributes significantly to microbial burden in early life. A number of studies have suggested differences in the early colonization patterns of infants who go on to develop allergic diseases. These studies strongly suggest that the pattern of colonization in the first weeks of life may influence the patterns of allergic disease development [7, 8]. These notions have been supported by observations that gut flora can influence local and systemic immune responses. There has been speculation that intestinal flora may influence the maturing precursor cells that circulate through the gut before they home to other tissues. This may explain how probiotic species can influence systemic immune responses and immunoglobulin (Ig) A production in distal sites, such as the respiratory tract. Thus, certain probiotics seem to influence the gut's allergen-stimulated inflammatory response and provide a barrier effect against antigens that might otherwise ultimately lead to systemic allergic symptoms (such as eczema). Together with reported clinical effects in early allergic disease, this has logically led to a growing interest in the role of probiotics in allergy prevention [1, 2].

### 1.2. Allergic Skin Conditions (Reactions) and Atopic Dermatitis (Eczema)

The literature on probiotic use in allergic skin reactions mainly includes experiments in AD (human and animal), AD-like skin lesions, and allergic contact dermatitis in animal experiments. And AD can be accepted as a prototypic disease for skin allergy reactions. 

AD is the most common chronic skin allergy reaction in children and adults, with a prevalence of 10% to 20% in population. Geographic location affects the prevalence of this disease, with the highest prevalence in the USA and Europe [9]. Important factors in the susceptibility to develop AD include a genetic basis and environmental factors. Eczema refers to a chronic or relapsing itchy skin inflammation with typical lesions and locations. Eczema is called atopic if it is associated with IgE demonstrated by either positive skin prick tests or elevated antigen-specific IgE antibodies. The term atopy refers to a genetic predisposition to become sensitized and to mount an IgE response to allergens. AD has been linked to food hypersensitivity, especially milk and egg proteins. However, 40%–60% of children with AD may not develop IgE sensitization [10]. The term eczema has been recently proposed, but, for practical purposes, both AD and eczema will be used in this paper.

There have been several proposed methods for classifying the severity of AD in various research studies mentioned in this paper, but only the SCORAD, established by the European Task Force on AD, has been validated for reproducibility and accuracy in assessing therapeutic response [9, 10]. The SCORAD combines objective measures, such as extent and severity of skin lesions, and subjective criteria, such as pruritus and sleep loss. Children with AD can be further classified as having mild, (≤25); moderate, (25–50); or severe, (≥50) disease based on their SCORAD scores.

### 1.3. What Are Probiotics?

Year 2013 marks the 106 year since Metchnikoff suggested that the consumption of lactic acid bacteria (LAB) may benefit the human host's immune system [55]. However, not until the mid 1960s did the term probiotic become the trend. The term probiotics means “for life” and is defined by the World Health Organization and the Food and Agriculture Organization of the United Nations as “live microorganisms which, when administered in adequate amounts as part of food, confer a beneficial health effect by producing gut microflora on the host.” These probiotics are mainly represented by LAB [56]. Simply, probiotics are ingested live microbes that can modify intestinal microbial populations in a way that benefits the host.

Probiotic intestinal flora contributes to microbial antigen exposure in early life and is one of the most abundant sources of early immune stimulation. Because allergic immune responses manifest early in life, there has been obvious interest in the potential benefits of modifying the gastrointestinal flora by using probiotic supplementation. However, the value of probiotics for primary prevention of these diseases is controversial [1, 2]. So far, there have been only several studies to address the role of probiotics in primary prevention of allergic skin conditions, with a reported suspicious reduction in the incidence of eczema. Since the role of probiotics in allergy prevention has remained controversial and there has been an urgent call for similar studies to address this further, this paper will try to highlight the role of probiotics in the therapy/prevention of allergic skin reactions and the future of this therapy. 

## 2. Mechanisms of Probiotics' Effects in Allergic Skin Conditions

Although the beneficial effects of probiotics on wide variety of atopic diseases have been suggested, little is known about how probiotics modulate the immune system, atopic disease development, and skin allergy reactions. Currently, only limited publications are available defining the effects of probiotics in murine or human models of AD and skin allergy reactions. Therefore, it is important to explore the effects of probiotics in these models [57]. In this section, experimental (animal) models and clinical studies showing mechanisms of probiotics' effects in skin allergy reactions and AD are being discussed [8, 58].

### 2.1. Maturing Gut Barrier: Probiotic Regulation in Intestinal Epithelium and Upregulation of Host Immune Responses

Recent data indicate that commensal intestinal microbiota represents a major modulator of intestinal homeostasis. Dysregulation of the symbiotic interaction between the intestinal microbiota and the mucosa may result in a pathological condition with potential clinical repercussions. For instance, it is shown that mice reared in germ-free conditions have underdeveloped immune systems and have no oral tolerance [6]. In contrast, pathogen-free mice are capable of reconstituting the bacterial flora with Bifidobacteria and tolerance development [59].

In addition to providing maturational signals for the gut-associated lymphoid tissue, probiotics balance the generation of pro- and anti-inflammatory cytokines in the gut. Some components of heat-treated LGG may have an ability to delay the onset and suppress the development of AD in NC/Nga mice, probably through a strong induction of IL-10 in intestinal lymphoid organs and systemic levels [14]. After probiotic consumption, decrease in fecal *α*-1 antitrypsin and serum TNF-*α* and changes in TGF-*β* and other cytokines point to downregulation of inflammatory mediators [18]. For instance, after a challenge study in infants allergic to cow's milk, fecal IgA levels were detected to be higher, and serum TNF-*α* levels were lower in the LGG-applied group compared with the placebo [32]. Similarly, another study by Kirjavainen et al. suggested that Bfdbm lactis Bb12 might modify gut microflora to alleviate early onset atopic eczema. And this modification was found to be compatible with reductions of serum TNF-*α* and fecal *α*-1-antitrypsin levels as well as an increase in fecal IgA level [60]. 

Moreover, probiotic bacteria may counteract the inflammatory process by stabilizing the gut microbial environment and the permeability barrier of the intestine, and by enhancing the degradation of enteral antigens and altering their immunogenicity [61]. This gut-stabilizing effect of probiotics could be explained by the improvement by probiotics of the immunological barrier of the intestine through intestinal IgA responses; see specifically [33, 62]. Oral treatment with probiotic Lctbs johnsonii NCC533 (La1) for a specific part of the weaning period was also shown to prevent the development of AD in model mice, NC/Nga, by modulating or accelerating the gut immune response with increased intestinal secretory IgA [63]. Consistent with these explanations, in children with food allergies, probiotics are shown to reverse increased intestinal permeability and to enhance frequently defective IgA responses [32, 64]. 

### 2.2. Immunomodulation: Th1/Th2 Balance, IgE Production, and Cytokines

In addition to maturing gut barrier, certain strains of Lactobacilli and Bifidobacteria modulate the production of cytokines by monocytes and lymphocytes and may divert the immune system in a regulatory or tolerant mode [59, 65]. Nonetheless, there are still some studies showing no significant effects of probiotics on either Th1 or Th2 cell responses to allergens. Although the cytokine stimulation profiles of different probiotic strains vary, the strains isolated from healthy infants mainly stimulate noninflammatory cytokines [66]. Therefore, it seems that changes in cytokine profiles induced by probiotics may be probiotic strain or site specific and dependent on the experimental system used. For instance, Lctbs reuteri induced proinflammatory and Th1 cytokines; Bfdbm bifidum/infantis and Lctbs lactis reduced Th2 cytokines [67]. 

Oral administration of LAB isolated from the traditional South Asian fermented milk “dahi” inhibits the development of AD in NC/Nga mice as well. Of the 41 strains tested from “dahi”, Lctbs delbrueckii subsp. lactis R-037 exhibited the greatest IL-12 induction, suggesting that it is a potent Th1 inducer [11]. Also, the antiallergic effects of one strain (T120) of LAB isolated from the Mongolian fermented milk using AD model mice (NC/Nga mice) were investigated. Strain T120 has already been identified as Enterococcus faecium, suppressed total IgE production, and induced IL-12 and IFN-*γ* production by splenocytes of NC/Nga mice. Furthermore, this strain enhanced the production of IL-10 by splenocytes, and activation of T regulatory (Treg) cells by strain T120 may inhibit atopic disease. In in vivo studies, intraperitoneal injection of strain T120 inhibited serum IgE elevation and AD symptoms in NC/Nga mice [12]. In another study, Lctbs plantarum strains from Kimchi were demonstrated to inhibit AD (house-dust mite-induced dermatitis) in NC/Nga mice. The three strains, CJLP55, CJLP133, and CJLP136, suppressed AD-like skin lesions and epidermal thickening. These same three strains decreased Th2 cytokines production such as IL-4 and IL-5 in lymph node cell cultures. The latter two, CJLP133 and CJLP136, increased IFN-*γ* secretion, while CJLP55 enhanced IL-10 production. These findings suggest that Lactobacilli isolated from Kimchi inhibit AD, probably by altering the balance of Th1/Th2 ratio or by inducing IL-10 production [68]. Similarly, Lctbs acidophilus strain L-55 suppressed the development of AD-like skin lesions induced by repeated application of TNCB in sensitized NC/Nga mice via a decrease in the serum total IgE level [69]. 

AD-like skin lesions were induced by sensitization to and repeated challenges with picrylchloride in the Th2-skewed NC/Nga mice strains. A new synbiotic, Lctbs casei subsp. casei together with dextran, reduces murine allergic reaction such as the development of AD-like skin lesions in NC/Nga mice. This synbiotic combination significantly decreased clinical skin severity scores induced by picryl chloride and total IgE levels in sera of NC/Nga mice [15]. Also, supplementation with KW3110 strain of LAB significantly attenuated the onset and exacerbation of AD-like skin lesions, accompanied by less mast cell infiltration and lower plasma IgE levels through its effects on IL-12 and IL-4 production in vitro [21]. Furthermore, oral administration of heat-killed Lctbs brevis SBC8803 ameliorates the development of dermatitis in AD model of NC/Nga mice. Eight-week-old male NC/Nga mice were sensitized by the topical application of picryl chloride to foot pads and shaved abdomens. Oral administration of Lctbs brevis SBC8803 significantly inhibited IgE production and ear swelling and suppressed the development of dermatitis in a dose-dependent manner. Immunosuppressive cytokines such as IL-10 and TGF-*β* production from Peyer's patch cells significantly increased in the treatment group, compared with the control group [22]. Consistently, oral supplementation with Lctbs rhamnosus CGMCC 1.3724 (LPR) in a study by Tanaka et al. has been demonstrated to prevent development of AD in NC/NgaTnd mice possibly by modulating local production of IFN-*γ* and plasma total IgE in skin biopsies, compared with untreated mice [19]. 

A decrease in the secretion of proinflammatory cytokines, IFN-*γ*, TNF-*α*, and IL-12, has been demonstrated. Consistently, in an experimental study, probiotic supplementation decreased the severity of allergic skin responses in allergen-sensitized pigs with a corresponding increase in IFN-*γ* expression [70]. Similarly, Pohjavuori et al. were able to demonstrate an increase of IFN-*γ* production in peripheral blood mononuclear cell in infants with AD treated with LGG instead of placebo [71]. Additionally, the improvement in AD severity in very young children with probiotic treatment was detected to be associated with significant increases in the capacity for Th1 IFN-*γ* responses and altered responses to skin and enteric flora. This effect was still evident 2 months after the supplementation was ceased [72].

Twelve human studies were included in a review, and 67% showed a positive association with TGF-*β*1 or TGF-*β*2 demonstrating protection against allergy-related outcomes in infancy and early childhood. High variability in concentrations of TGF-*β* was noted between and within studies, with some of it explained by maternal history of atopy or by consumption of probiotics. Human milk TGF-*β* appears to be essential in developing and maintaining appropriate immune responses in infants and may provide protection against adverse immunological outcomes, corroborating findings from experimental animal studies. In a study, the aim was to evaluate the effect of probiotic supplementation on the immunological composition of breast milk and colostrum in relation to sensitization and eczema in babies. Supplementation of probiotics during pregnancy was associated with low levels of TGF-*β*2 and slightly increased levels of IL-10 in colostrum. Infants receiving breast milk with low levels of TGF-*β*2 were less likely to become sensitized, and it was likely to find possibly less IgE-associated eczema in breast-fed infants during their first 2 years of life [44]. However, another trial by Boyle et al. showed that LGG treatment during pregnancy (prenatal) for the prevention of eczema was associated with decreased breast milk soluble CD14 and IgA levels, not TGF-*β* [47]. The difference between these studies depends on probiotic species, which may affect the immunological composition of breast milk. 

### 2.3. Anti-Inflammatory Effects: Their Effects on Serum Inflammatory Parameters

The anti-inflammatory effect of probiotics has been attributed to increased production of IL-10 by immune cells in the lamina propria, Peyer's patches, and the spleen of treated animals [66, 67, 73, 74]. Oral administration of LGG resulted in elevated IL-10 concentrations in atopic children, indicating that specific probiotics may have anti-inflammatory effects in vivo and may possibly enhance regulatory or tolerance-inducing mechanisms as well. In a review of the evidence from randomized controlled trial (RCTs) by Betsi et al. about probiotics for the treatment or prevention of AD, the results of 13 relevant randomized (placebo)-controlled trials were reviewed: 10 of which evaluated probiotics as treatment and 3 for prevention of AD. In four of those RCTs, clinical improvement was associated with a change in some inflammatory markers [75]. 

A study by Woo et al. evaluated the effect of Lctbs sakei supplementation in children with atopic eczema-dermatitis syndrome (AEDS). In this study, compared with placebo, probiotic administration was associated with lower pretreatment-adjusted serum levels of chemokines such as CCL17 and CCL27, which were significantly correlated with SCORAD total score [36]. 

Probiotic-induced chronic low-grade inflammation characterized by elevation of CRP, IgE, IgA, and IL-10 was shown in some studies, with the changes being typically observed in helminth infection-associated induction of regulatory mechanisms. The association of increased CRP with a decreased risk of eczema at 2 years of age in allergy-prone children supports the view that chronic, low-grade inflammation protects from eczema. The findings emphasize the role of chronic microbial exposure as an immune modulator protecting from allergy [40]. 

Primary administration of Lctbs johnsonii NCC533 (La1) in the weaning period suppressed the elevation of proinflammatory cytokines and CD86 gene expression levels in skin lesions of NC/Nga model mice. The suppression of proinflammatory cytokines such as IL-8/-12/-23 and CD86 expression by primary administration of La1 may significantly contribute to the inhibitory effects on the skin lesions like AD [76].

In a study by Rosenfeldt et al., 2 probiotic Lctbs strains (lyophilized Lctbs rhamnosus 19070-2 and Lctbs reuteri DSM 122460) were given in combination for 6 weeks to 1- to 13-year-old children with AD. During active treatment, serum eosinophil cationic protein (ECP) levels significantly decreased. A combination of Lctbs rhamnosus and Lctbs reuteri was beneficial in the management of AD, and the effect was more pronounced in atopic eczema patients [27]. Another study that was conducted by Brouwer et al. showed, during Lctbs species supplementation, that a moderate but significant reduction in soluble ECP levels was found. ECP, a cytotoxic protein released from activated eosinophils, has been used to monitor disease activity in AD. Thus, soluble ECP might be a more sensitive marker in acute exacerbations of the eczema than a marker of disease activity per se [52]. 

### 2.4. Development of Tolerogenic Dendritic Cells

Selected species of the Bfdbm genus were demonstrated to prime in vitro cultured neonatal dendritic cells (DCs) to polarize T cell responses and may, therefore, be used as candidates in primary prevention of allergic diseases. Bfdbm bifidum was found to be the most potent polarizer in in vitro-cultured DCs to drive Th1-cell responses involving increased IFN-*γ*-producing T-cells concomitant with reduction of IL-4-producing T-cells [77]. In addition, T-cells stimulated by Bfdbm bifidum matured DCs as producers of more IL-10 [78]. Moreover, Lctbs rhamnosus, a member of another genus of probiotic bacteria, modulates DCs functions to induce a novel form of T-cell hyporesponsiveness [79]. Lctbs reuteri/casei have been also shown to prime monocyte-derived DCs through the C-type lectin DC-specific intercellular adhesion molecule 3-grabbing nonintegrin (DC-SIGN) to drive the development of Treg cells [80]. These Treg cells produce increased levels of IL-10 and are capable of inhibiting the proliferation of bystander T-cells. This study suggests that the targeting of DC-SIGN by certain probiotic bacteria might explain their beneficial effect in the treatment of a number of inflammatory diseases, including AD.

### 2.5. Immunoregulation by T Regulatory (Treg) Cells

Generation of CD4+/Foxp3+ Treg cells by probiotics administration suppresses immune and allergic disorders. Recently, two studies reported that oral administration of a certain probiotic strain could increase Foxp3+ Tregs [81]. It is known that the lower percentage of epidermal or dermal Foxp3+ cells in eczematous dermatitis might contribute to their pathogenesis [82]. The strain T120 of LAB was shown to be able to inhibit atopic disease in NC/Nga mice through enhanced production of IL-10 by splenocytes and activation of Treg cells [12]. 

In a recent study, a mixture of probiotics (Lctbs acidophilus, Lctbs casei, Lctbs reuteri, Bfdbm bifidum, and Streptococcus thermophilus) was identified, and it upregulates CD4+/Foxp3+ Treg cells. Administration of the probiotics mixture induced both T-cells and B-cells hyporesponsiveness and downregulated Th1, Th2, and Th17 cytokines [81, 83]. It also induced generation of CD4+/Foxp3+-Tregs from the CD4+/25 population and increased the suppressor activity of naturally occurring CD4+/25+-Tregs. Conversion of T cells into Foxp3+ Tregs is directly mediated by regulatory DCs that express high levels of IL-10 and TGF-*β*. In a murine AD model, treatment with this probiotic mixture significantly inhibited the clinical symptoms of AD progression by reducing IgE levels (total and specific IgE levels), infiltrated lymphocytes and granulocytes, and levels of AD-associated cytokines [81]. 

Lctbs casei treatment enhanced the frequency of FoxP3+-Tregs in the skin and increased the production of IL-10 by CD4+/25+-Tregs cells in skin-draining lymph nodes of hapten-sensitized mice. These data demonstrate that orally administered Lctbs casei efficiently alleviate T-cell-mediated skin inflammation without causing immune suppression, via mechanisms that include control of CD8+-effector T-cells and involve regulatory CD4+-T-cells. Lctbs casei may, thus, represent a probiotic of potential interest for immunomodulation of T-cell-mediated allergic skin diseases in human beings [25]. 

In sensitized BALB/c mice, skin inflammation was induced by topical allergen application. Escherichia coli Nissle 1917 was administered orally in a preventative manner. Oral Escherichia coli Nissle administration improved allergen-induced dermatitis dose dependently. In parallel, a reduction of epidermal thickness and infiltrating immune cells together with an enhanced number of Foxp3 (+) cells and a trend of increased IFN-*γ*, IL-10, and TGF-*β* expression levels was detected in eczematous skin. Our findings indicate that Escherichia coli Nissle alters the local allergen-induced immune response by increase of Foxp3 (+) cells and by favoring an immunoregulatory cytokine pattern [26]. 

### 2.6. Lymphocyte Subpopulations

Several studies reveal that the probiotics differently modulate peripheral blood immune parameters in healthy subjects and patients with AD. 

Gerasimov et al. conducted a study to assess the clinical efficacy and impact of Lctbs acidophilus and Bfdbm lactis with fructooligosaccharide on peripheral blood lymphocyte subsets in preschool children with moderate-to-severe AD. The percentage of CD4 and the percentage and absolute count of CD25 decreased; and the percentage and absolute count of CD8 increased significantly in the probiotic group at week 8, compared with placebo. They found a significant correlation between CD4 percentage, CD25 percentage, CD25 absolute count, and SCORAD values in the probiotic group at week 8. The administration of a probiotic mixture and fructooligosaccharide was correlated with significant clinical improvement in children with AD, with corresponding lymphocyte subpopulation changes in peripheral blood [46]. 

Also in other mice studies, contact hypersensitivity to the hapten 2,4-dinitrofluorobenzene, a model of allergic contact dermatitis mediated by CD8+-cytotoxic T-lymphocytes and controlled by CD4+-Treg cells, was studied. Daily oral administration of fermented milk containing Lctbs casei or Lctbs casei alone decreased skin inflammation by inhibiting the priming/expansion of hapten-specific IFN-*γ*-producing CD8+-effector T-cells. This study provides the first evidence that oral administration of Lctbs casei can reduce antigen-specific skin inflammation by controlling the size of the CD8+-effector pool [24]. Nevertheless, oral treatment with the probiotic bacteria Lctbs casei alone alleviated antigen-specific skin inflammation mediated by either protein-specific CD4+-T-cells or hapten-specific CD8+-T-cells in hapten-sensitized mice. In the model of CD8+-T-cell-mediated skin inflammation, reproducing allergic contact dermatitis in human beings, inhibition of skin inflammation was due to decreased CD8+-effector T-cells recruitment into the skin during the elicitation (i.e., symptomatic) phase of contact hypersensitivity [25].

### 2.7. Toll-Like Receptor (TLR) Stimulation

A number of experiments indicate that infectious agents can promote protection from ADs through mechanisms independent of their constitutive antigens, leading to stimulation of non-antigen-specific receptors such as TLRs. A family of pattern-recognition receptors such as TLRs on gut lymphoid and epithelial cells mediates innate immune responses to bacterial molecular patterns and, thereby, orchestrates acquired immunity. The transient protection offered by probiotics against IgE-associated allergic diseases is based on stimulation of TLRs, which produce mediators such as IL-6; these further induce IgA differentiation from naive B-cells. These events were shown to occur after probiotic administration to infants with eczema, as well as in infants who showed increased levels of serum CRP, IL-10, and IgE at the age of 6 months [40]. This probiotic-induced low-grade inflammation was characterized by elevation of CRP, IgE, IgA, and IL-10, with the changes being typically observed in helminth infection-associated induction of regulatory mechanisms. Moreover, the association of increased CRP with a decreased risk of eczema at 2 years of age in allergy-prone children supports the view that chronic, low-grade inflammation protects from eczema. The findings emphasize the role of chronic microbial exposure as an immune modulator protecting from allergy through activation of Treg cells. Consistently, LAB species such as Bfdbm bifidum/infantis and Lctbs salivarius were shown to be capable of activating TLR-2 [84]. In summary of the various effects of different probiotic strains in skin allergy reactions, local influences of probiotics potentially include reduction of gut permeability and systemic penetration of antigens, increased local IgA production, and alteration of local inflammation or tolerance induction. Some possible systemic effects consist of anti-inflammatory effects mediated by Toll-like receptors (TLRs), T-helper 1 (Th1) skewing of responses to allergens, and activation of tolerogenic dendritic cells (DCs), in addition to Treg cell production [1, 2, 85].

## 3. Experimental (Animal Model) and Clinical (Human) Studies Showing the Role of Probiotics in the Prevention and Treatment of Allergic Skin Conditions

The increased prevalence of allergic diseases is nowadays defined as an epidemic. AD is known as the earliest of these conditions, and it might act as an indicator for the development of IgE- or non-IgE-mediated allergic manifestations. Thus, being aware of possible measures, such as probiotic use, to prevent and/or heal atopic disease is essential for the practicing allergy specialist. Here, their role in the prevention/therapy of AD and allergic skin conditions under the recent literature gathered from Medline and Pubmed is discussed. 

### 3.1. Experimental Studies Showing the Role of Probiotics in the Prevention/Treatment of Allergic Skin Conditions

Over the several decades, animal models of AD and skin allergy reactions have received increasing attention. These models include NC/Nga mice, a hapten-induced mouse model, and transgenic and knockout mouse models. Although the pathogenesis of skin inflammation elicited in these models is not quite the same, it is pertinent to ask what these animal models really tell us about the pathogenesis and possible therapies for the disease. NC/Nga mice may yield information relevant to the dissection of the crucial components of the pathophysiology of skin allergy reactions and AD rather than the assessment of potentially therapeutic agents for their treatment. And this hapten-induced mouse model has been mostly used and created by repeated applications of 2,4,6-trinitrochlorobenzene (TNCB), that is, a simple and reproducible one. This model offers several advantages over others: by changing hapten and the mouse strain used, various types of chronic inflammation, probably reflecting heterogeneity in clinical presentation of skin allergy reactions and AD, can be induced. This model is also of enormous value in its high reproducibility as well as the ease of quantitative assessment by measuring ear thickness [57, 86]. 

Probiotic strains have been reported to have the ability to control allergic and inflammatory diseases. Here, some of the studies performed on experimental murine models of AD and AD-like lesions showing the role of probiotics will be discussed (the various effects of different probiotic strains, referred to in this paper, on AD, AD-like skin lesions, and allergic contact dermatitis in experimental (animal) studies are shown in Table 1 as well).

#### 3.1.1. Murine Models of AD Induced by House-Dust Mite Sensitization

Oral administration of Lctbs delbrueckii subsp. lactis R-037 isolated from the traditional South Asian fermented milk “dahi” inhibited the development of AD in NC/Nga mice [11]. In addition, the antiallergic effect of one strain (T120) of LAB isolated from the Mongolian fermented milk using AD model mice (NC/Nga mice) was investigated. And in in vivo studies, intraperitoneal injection of strain T120 subdued AD symptoms in NC/Nga mice [12]. In another study, Lctbs plantarum strains from Kimchi were investigated for their capacity to inhibit AD (house dust mite-induced dermatitis) in NC/Nga mouse. The three strains, CJLP55, CJLP133, and CJLP136, suppressed AD-like skin lesions and epidermal thickening [13, 23, 87].

Ingestion of heat-treated LGG was shown to prevent development of AD of NC/Nga mice in a study. Maternal and infant mice were fed with food containing or not containing heat-treated LGG during pregnancy and breastfeeding, and after weaning. Administration of food containing heat-treated LGG inhibited the onset and development of atopic skin lesions, accompanied by smaller numbers of mast cells and eosinophils in the affected skin sites [14, 21]. Moreover, a new synbiotic, Lctbs casei subsp. casei together with dextran reduced murine allergic reaction such as the development of AD-like skin lesions developed by Dermatophagoides pteronyssinus crude extract in NC/Nga mice. This combination significantly decreased clinical skin severity scores and total IgE levels in sera of NC/Nga mice [15]. Nevertheless, administration of LGG to puppies appeared to reduce immunologic indicators (allergen-specific IgE) of AD, although no significant decrease in clinical signs (dermatitis and pruritus) was detected. In this study, the efficacy of the probiotic LGG for the alleviation or prevention of clinical signs of AD in genetically predisposed dogs (2 adult Beagles with severe AD and 16 puppies) was evaluated. LGG was administered to the bitch during the second pregnancy and to the puppies of the second litter from 3 weeks to 6 months of age. Both litters were epicutaneously sensitized to Dermatophagoides farinae [16, 17]. 

In a recent study, the inhibitory effect of Bacillus subtilis on AD was studied too. The effects of continuous oral administration of Bacillus subtilis for 4 weeks on the development of AD induced by Dermatophagoides farinae body antigen in NC/Nga mice were evaluated using 4 groups of mice. Histopathological examination results revealed significant differences suggesting that continuous oral administration of Bacillus subtilis can be effective in alleviating the development of skin lesions induced by Dermatophagoides in NC/Nga mice [88].

#### 3.1.2. Murine Models of AD-Like Skin Lesions Induced by Trinitrochlorobenzene Sensitization

In a study, Lctbs acidophilus strain L-55 suppressed the development of AD-like skin lesions induced by repeated applications of TNCB in sensitized NC/Nga mice. The increase of dermatitis score and ear swelling was also inhibited by strain L-55. Scratching behavior observed in the back and ears was inhibited by strain L-55 as well. Furthermore, strain L-55 also caused an inhibition of histological changes induced by repeated applications of TNCB [18, 89].

Oral treatment with probiotic Lctbs johnsonii NCC533 (La1) during the specific part of the weaning period prevented the development of AD in model mice, NC/Nga. In a similar study, La1 was also administered orally to the La1 group from 20 to 22 days after birth. After the induction of skin lesions in 6-week-old mice, the expression of genes supposedly involved in AD was evaluated. Gene expression of the proinflammatory cytokines such as IL-8, IL-12, and IL-23 was significantly enhanced in the lesional skin of the control group by the induction of the lesion, whereas gene expression of those in the La1 group was not elevated. Moreover, the La1 group showed a significantly lower gene expression of CD86 in Peyer's patches and mesenteric lymph nodes than the control group. The suppression of proinflammatory cytokines and CD86 expression by primary administration of La1 may significantly contribute to the inhibitory effect on the skin lesions [20, 90, 91].

Oral supplementation with Lctbs rhamnosus CGMCC 1.3724 (LPR) prevented development of AD in NC/NgaTnd mice possibly by modulating local production of IFN-*γ* in a study. Pregnant NC/NgaTnd mice were orally treated with the probiotic strain LPR, which was followed by treatment of pups until 12 weeks of age. LPR-treated mice exhibited significantly lower clinical symptoms of dermatitis and reduced scratching frequency, compared with untreated mice. The protective effect was also observed when mice started to be treated at weaning time (5 weeks of age) even with limited supplementation period of 2 weeks. However, treatment of mice with the probiotic starting 1 week after the onset of the disease (8 weeks of age) had limited effects [19]. 

#### 3.1.3. Murine Models of AD-Like Skin Lesions Induced by Picryl Chloride Sensitization

AD-like skin lesions were induced by sensitization to and repeated challenges with picryl chloride in the Th2-skewed NC/Nga mouse strain. A new synbiotic, Lctbs casei subsp. casei together with dextran reduced murine allergic reaction such as the development of AD-like skin lesions in NC/Nga mice. This synbiotic combination significantly decreased clinical skin severity scores induced by picryl chloride, similar to dust mite sensitization, in NC/Nga mice [15]. Supplementation with KW3110 strain of LAB significantly attenuated the onset and exacerbation of AD-like skin lesions, accompanied by less mast cell infiltration [16].

Oral administration of heat-killed Lctbs brevis SBC8803 ameliorated the development of dermatitis in AD model NC/Nga mice. Eight-week-old male NC/Nga mice were sensitized by the topical application of picryl chloride to foot pads and shaved abdomens. These mice were boosted with picryl chloride by topical application onto the ears once a week for 9 weeks. The mice (*n* = 10 per group) were fed a diet containing 0%, 0.05%, or 0.5% of heat-killed Lctbs brevis from 2 weeks before the first sensitization to the end of the study. Oral administration of Lctbs brevis significantly inhibited ear swelling and suppressed the development of dermatitis in a dose-dependent manner [22].

#### 3.1.4. Murine Models of Allergic Contact Dermatitis Induced by Dinitrofluorobenzene Sensitization

The aim of a few studies was to examine whether Lctbs casei could affect antigen-specific CD8+ -T-cell-mediated skin inflammation. In a study by Chapat et al., contact hypersensitivity to the hapten 2,4-dinitrofluorobenzene, a model of allergic contact dermatitis mediated by CD8+-cytotoxic T-lymphocytes and controlled by CD4+-Treg cells, was used. This study provided the first evidence that oral administration of Lctbs casei could reduce antigen-specific skin inflammation by controlling the size of the CD8+-effector pool [24]. Similarly, oral treatment with the probiotic bacteria Lctbs casei alone alleviated antigen-specific skin inflammation mediated by either protein-specific CD4+-T-cells or hapten-specific CD8+-T-cells in hapten-sensitized mice. In the model of CD8+-T-cell-mediated skin inflammation, which reproduces allergic contact dermatitis in human beings, inhibition of skin inflammation by Lctbs casei was due to attenuation of the recruitment of CD8+-effector T-cells into the skin during the elicitation (i.e., symptomatic) phase of contact hypersensitivity. These data demonstrate that orally administered Lctbs casei efficiently alleviate T-cell-mediated skin inflammation without causing immunosuppression [25].

In sensitized BALB/c mice, skin inflammation was induced by topical allergen application. Escherichia coli Nissle 1917 was administered orally in a preventative manner and it improved allergen-induced dermatitis dose dependently, consistent with a reduction of epidermal thickness that was detected in eczematous skin [26].

Lctbs sakei probio-65 that was isolated from Kimchi, a traditional Korean fermented food, was found to be effective in reducing allergic dermatitis in chemical allergen- (1-chloro-2,4-dinitrobenzene-) induced mice as well [68, 92].

### 3.2. Clinical (Human) Studies Showing Probiotics' Effects in Allergic Skin Conditions including Eczema

Mostly reported clinical (human) studies showing probiotics' effects in skin allergy reactions have been related to AD (eczema). Here, probiotics' effects in human AD are being discussed according to the IgE-sensitized (atopic) versus non-IgE-sensitized (nonatopic) eczema groups (the various effects of different probiotic strains, referred to in this paper, on allergic skin conditions including AD in clinical (human) studies are shown in Table 2).

*Is There Any Difference between IgE-Sensitized (Atopic) and Non-IgE-Sensitized (Nonatopic) Eczema Groups?* A number of studies could only relate probiotic benefits to a certain subset of AD patients. In support of the efficacy of probiotics in IgE-sensitized children, some other studies also demonstrated comparable results as well. In brief, treatment with Lctbs rhamnosus for the first 2 years of life was associated with a significant reduction in the prevalence of any IgE-associated eczema by about a half [4]. Another study demonstrated that LGG alleviated atopic eczema/dermatitis syndrome symptoms in IgE-sensitized infants [18]. In food-sensitized atopic children, the efficacy of the probiotics such as Lctbs rhamnosus and Bifidobacterium (Bfdbm) lactis was demonstrated too [28]. This effect was more pronounced in patients with a positive skin prick test and increased IgE levels.

Yet, some other studies failed to demonstrate that the severity and frequency of AD were decreased with the supplementation of probiotics, regardless of their IgE sensitization status. For instance, Boyle et al. and others could not show any effect even of LGG in infants with AD [47, 48]. A few meta-analyses also could not confirm that IgE sensitization was indeed a factor in determining the efficacy of probiotics in atopic children. However, the heterogeneity between studies may be attributable to probiotic strain-specific effects and other factors as well, meaning that some probiotic strains may still have a therapeutic role in eczema [1, 2].

#### 3.2.1. IgE-Sensitized (Atopic) Eczema Therapy and Prevention

Recently was published one of the largest studies by Viljanen et al. to date that compared LGG or a probiotic mix (LGG, Lctbsrhamnosus LC705, Bfdbm breve Bb99, and Propionibacterium freudenreichii ssp. shermanii JS) with placebo. In that study, 230 Finnish children with AD were treated for 4 weeks with LGG, a mixture of four probiotic strains, or placebo. With supplementation of probiotics (LGG), Viljanen et al. found significant improvement on the SCORAD index only in “IgE-sensitize cow's milk-allergic infants of the AEDS.” Only in the subgroup of IgE-sensitized children did the LGG group show a greater reduction in SCORAD than the placebo group, but this effect could have been due to a higher baseline score in this subgroup. There was no difference between the groups at the end of the 4-week therapy, and 4 weeks after therapy was discontinued. Contrary to what would be expected, improvement was seen 4 weeks after discontinuation of therapy rather than during treatment [93]. Rosenfeldt et al. from Denmark in a study demonstrated that 2 lyophilized probiotic Lctbs strains (lyophilized Lctbs rhamnosus 19070-2 and Lctbs reuteri DSM 122460) were given in combination for 6 weeks to 1- to 13-year-old (mean age, 5.2 years) children with AD. This study used 2 different Lctbs species in older children. A combination of these was beneficial in the management of AD. Statistically significant improvement in SCORAD score was seen only in a subset of children with positive skin prick test results and elevated IgE levels [27]. Another study by Sistek et al. showed the efficacy of the probiotics Lctbs rhamnosus and Bfdbm lactis in food-sensitized children [28].

A study by a Finnish group used the same probiotic mixture with prebiotics. Kukkonen et al. in a trial using probiotic mix (Lctbs rhamnosus GG, Lctbs rhamnosus LC705, Bfdbm breve Bb99; and Propionibacterium freudenreichii ssp. shermanii JS) and prebiotic galactooligosaccharides demonstrated that the prevention of atopic eczema in high-risk Finnish infants is possible by modulating the infants' gut microbiota with probiotics and prebiotics. Probiotic treatment compared with placebo reduced IgE-associated (atopic) diseases. Probiotic treatment also reduced eczema and atopic eczema [29, 94]. In 2009, in a study by Kuitunen et al., 1223 Finnish mothers were randomized with infants at high risk for allergy to receive the same probiotic mixture (2 Lactobacilli, Bifidobacteria, and Propionibacteria) or placebo during the last month of pregnancy, and their infants were to receive it from birth until the age of 6 months. Infants also received a prebiotic galactooligosaccharide or placebo. At 5 years, the cumulative incidence of allergic diseases (eczema, food allergy, allergic rhinitis, and asthma) and IgE sensitization were evaluated. Frequencies of allergic and IgE-associated allergic disease and sensitization in the probiotic and placebo groups were similar. However, less IgE-associated allergic diseases occurred in cesarean-delivered children receiving probiotics. No allergy-preventative effect that extended to the age of 5 years was achieved with perinatal supplementation of probiotic bacteria to high-risk mothers and children. It conferred protection only to cesarean-delivered children [30].

Similarly, Abrahamsson et al. could not confirm a preventative effect of probiotics (Lctbs reuteri ATCC 55730) on infant eczema in a recently published study. However, they observed that the treated infants had less IgE-associated eczema at 2 years. Moreover, skin prick test reactivity was also less common in the treated group than in the placebo group, but this difference reached significance only for infants with allergic Swedish mothers [31].

In summary, all of these studies taken together demonstrate that probiotics might not be effective and/or therapeutic for all children with AD, but they offer benefits to a subset of IgE-sensitized children. 

#### 3.2.2. Non-IgE-Sensitized (Nonatopic) Eczema Therapy and Prevention

Until now, several clinical studies have been published and have focused on the use of probiotics for therapy and primary prevention of atopic diseases. To date, the results of at least 15 prospective preventative studies with different Lctbs or Bfdbm strains (or mixture) in children at high risk for allergic diseases have been published. 

The first study in the literature by Isolauri et al. analyzed a benefit of LGG in mild AD disease in 1997. They observed 27 exclusively breastfed infants (median age, 4–6 months) with mild AD (median SCORAD score of 16), receiving extensively hydrolyzed whey formula with (LGG or Bfdbm strain) or without probiotics (placebo) for 8 weeks. They showed a reduction in the SCORAD by 15 points (from 16 to 1) for the LGG and by 16 points (from 16 to 0) for the Bfdbm arm, as compared with a reduction of 2–6 points (from 16 to 13–4) in the placebo arm. However, one month after therapy, SCORAD scores were comparable with those of placebo. Therefore, the probiotic effect was limited to acceleration of improvement in infants with mild disease [3]. The same investigators subsequently published 2 additional studies. One of these studies compared LGG with Bfdbm lactis Bb-12, both of which showed a significant improvement in SCORAD score over placebo. However, after 6 months, the median SCORAD score was zero in all groups, again suggesting that the effect is limited to rapid initiation of improvement [95]. The other study underlined the importance of viability for probiotic species. The use of heat-inactivated LGG resulted in adverse gastrointestinal symptoms with diarrhea, and study recruitment was halted. They concluded that supplementation of infant formulas with viable but not heat-inactivated LGG was found to be a potential approach for the management of atopic eczema and cow's milk allergy [96].

In an earlier study by Viljanen et al., probiotics have been suggested to be useful in children with AEDS. In 2010, a study by Woo et al. was performed to assess the clinical effect of Lctbs sakei supplementation in children with AEDS. In that study, children who aged 2 to 10 years with AEDS with a minimum SCORAD score of 25 were randomized to receive either daily Lctbs sakei KCTC 10755BP or daily placebo supplementation for 12 weeks. At week 12, SCORAD total scores adjusted by pretreatment values were lower after probiotic treatment than after placebo treatment. There was a 31% improvement in mean disease activity with probiotic use compared with a 13% improvement with placebo use. Therefore, significant differences in favor of probiotic treatment were also observed in proportions of patients achieving improvement of at least 30% and 50%. Interestingly, clinical improvement in this study was not just observed in the subgroup of IgE-sensitized children, contrary to the Viljanen et al. study, but it was also regardless of IgE sensitization [36]. Weston et al. from Australia published their experience with using Lctbs fermentum VRI-003 PCC for 8 weeks in 53 infants with AD. After 16 weeks, the probiotic group had significant reduction of SCORAD scores, while the placebo group did not. Lctbs fermentum caused a significant reduction in SCORAD scores. Although the change in SCORAD score from baseline in the probiotic group was significant, the difference between the probiotic and placebo groups did not reach significance by week 16 [37]. In a study by Hoang et al., they followed 14 cases of pediatric patients (ages of 8 months to 64 months) with a history of resistant eczema for a period of at least 6 months. All of these children received Lctbs rhamnosus cell lysate daily as an immunobiotic supplement. The results of this open-label nonrandomized clinical observation showed a substantial improvement in quality of life, skin symptoms, and day- and night-time irritation scores in children with the supplementation of Lctbs rhamnosus lysate. There were no intolerance or adverse reactions observed in these children. Lctbs rhamnosus cell lysate may, thus, be used as a safe and effective immunobiotic for the treatment and prevention of childhood eczema [38]. Bfdbm breve has been reported by Hattori et al. to improve cutaneous symptoms of AD patients. Fifteen children with AD who had Bfdbm-deficient microflora were selected for this study. Eight subjects in the Bifidobacteria-administered group were given oral administration of lyophilized Bfdbm breve M-16V strain. In the Bifidobacteria-administered group, the proportion of Bfdbm in the fecal microflora was increased, and the proportion of aerobic bacteria was decreased after 1 month of administration. Furthermore, significant improvement of allergic symptoms (in cutaneous symptoms and total allergic scores) was also observed in the Bifidobacteria-administered group. The tendency of allergic symptom improvement was remarkable compared with the control group; however, there was no correlation between changes in fecal microflora and allergic symptoms [39].

The Finnish study of Kalliomäki et al. was the first report to describe that the frequency of AD in the probiotic group was half that of the placebo. This hallmark study demonstrated that administration of LGG for 1 month before and 6 months after birth to their infants was associated with a significant reduction in the cumulative incidence of eczema during the first 7 years of life. The effect of probiotics on preventing AD has been demonstrated in infants of the Finnish pregnant mothers with a strong family history of eczema, allergic rhinitis, or asthma. The frequency of developing AD in the offspring was significantly reduced by 2, 4, and 7 years, by 50%, 44%, and 36%, respectively. But, there were no preventative effects on atopic sensitization and onset of respiratory allergic diseases [4].

Wickens et al. studied a differential effect of 2 probiotics in the prevention of eczema and atopy. Infants receiving Lctbs rhamnosus had a significantly reduced risk of eczema, compared with placebo, but this was not the case for B animalis subsp. lactis. In a double-blind, randomized placebo-controlled trial of infants at risk of allergic disease, pregnant women were randomized to take Lctbs rhamnosus HN001, Bfdbm animalis subsp. lactis strain HN019, or placebo daily from 35 weeks of gestation until 6 months if breastfeeding, and their infants were randomized to receive the same treatment from birth to 2 years (*n* : 474). Infants receiving Lctbs rhamnosus had a significantly reduced risk of eczema compared with placebo, but this was not the case for Bfdbm animalis subsp. lactis. There was no significant effect of Lctbs rhamnosus or Bfdbm animalis subsp. lactis on atopy. Lctbs rhamnosus (72%) was more likely than Bfdbm animalis subsp. lactis (22.6%) to be present in the feces at 3 months, although detection rates were similar by 24 months. The authors found out that supplementation with Lctbs rhamnosus, but not Bfdbm animalis subsp. lactis, substantially reduced the cumulative prevalence of eczema, but not atopy, by 2 years [34].

In a randomized double-blind study by Marschan et al., probiotic bacteria (Lctbs rhamnosus GG (ATCC 53103), Lctbs rhamnosus LC705, Bfdbm breve Bb99, and Propionibacterium freudenreichii ssp. Shermanii JS) or placebo had been given for 1 month before delivery to mothers and for 6 months to infants with a family history of allergy. Infants receiving probiotic bacteria had higher plasma levels of CRP, total IgA, total IgE, and IL-10 than infants in the placebo group. Increased plasma CRP level at the age of 6 months was associated with a decreased risk of eczema and with a decreased risk of allergic disease at the age of 2 years, when adjusted with probiotic use. The association of CRP with a decreased risk of eczema at 2 years of age in allergy-prone children supports the view that chronic, low-grade inflammation protects from eczema. Probiotic-induced low-grade inflammation was characterized by elevation of IgE, IgA, and IL-10, the changes typically observed in helminth infection-associated induction of regulatory mechanisms [40].

In the Panda study of Niers et al. administered was a mixture of probiotic bacteria (Bfdbm bifidum W23, Bfdbm lactis W52, and Lactococcus lactis W58; Ecologic Panda) for 6 weeks prenatally to mothers of high-risk children and to their offspring for the first 12 months of life. Although cumulative incidence of atopic eczema and IgE levels were similar in both treated and placebo groups, the parental reported eczema was significantly lower during the first 3 months of life in infants receiving probiotics. This particular combination of probiotic bacteria showed a preventative effect on the incidence of eczema in high-risk children, which seems to be sustained during the first 2 years of life. In addition to the previous studies, the preventative effect appeared to be established within the first 3 months of life in this study [41].

In a trial by Kim et al., 112 pregnant women with a family history of allergic diseases received a mixture of Bfdbm bifidum BGN4, Bfdbm lactis AD011, and Lctbs acidophilus AD031, starting at 4–8 weeks before delivery and continuing until 6 months after delivery. The cumulative incidence of eczema during the first 12 months was reduced significantly in the probiotic group; however, there was no difference in serum total IgE level or the sensitization against food allergens between the two groups. Prenatal and postnatal supplementation with a mixture of probiotics is an effective approach in preventing the development of eczema in infants at high risk of allergy during the first year of life [42].

In a randomized, double-blind trial by Dotterud et al., probiotics were given to pregnant women to prevent allergic diseases. In this study, children from a nonselected maternal population and women received probiotic milk or placebo from 36 weeks of gestation to 3 months postnatally during breastfeeding. The probiotic milk contained Lctbs rhamnosus GG, Lctbs acidophilus La-5, and Bfdbm animalis subsp. lactis Bb-12. At 2 years of age, all children were assessed for atopic sensitization, AD, asthma, and allergic rhinoconjunctivitis. Probiotics given to the nonselected mothers reduced the cumulative incidence of AD, but they had no effect on asthma or atopic sensitization [43].

Böttcher et al.'s study demonstrated that Lctbs reuteri supplementation during pregnancy is associated with reduced risk of sensitization during infancy. Swedish pregnant women were treated with Lctbs reuteri (*n* : 54) or placebo (*n* : 55) from gestational week 36 until delivery. The infants were followed prospectively for 2 years regarding development of eczema and sensitization as defined by a positive skin prick test and/or circulating allergen-specific IgE antibodies at 6, 12, and 24 months of age [44].

Of note, another recently published Swedish study demonstrated that administration of Lctbs casei F19 during weaning significantly reduced the incidence of eczema, indicating that proper timing of the probiotic intervention is a critical factor. That study also supports the notion that there is more than a single window of opportunity to manage allergic diseases. That study, moreover, evaluated the effects of feeding with Lctbs F19 during weaning period on the incidence of eczema and Th1/Th2 balance. In this intervention trial by West et al., infants were fed cereals with (*n* : 89) or without Lctbs F19 (*n* : 90) from 4 to 13 months of age. The cumulative incidences of eczema at 13 months 11% and 22% in the probiotic and placebo groups, respectively were (*P* : <0.05). At 13 months of age, the IFN-*γ*/IL-4 mRNA ratio was significantly higher in the probiotic group compared with the placebo group. The higher Th1/Th2 ratio in the probiotic group compared with the placebo group suggests enhancing effects of Lctbs F19 on the T-cell-mediated immune response. In contrast, there were no differences between groups in serum IgE concentrations. As a result, feeding Lctbs F19 during weaning could be an effective tool in the prevention of early manifestation of allergy such as eczema [35].

Oral administration of probiotic Escherichia coli after birth in the early postnatal period by Lodinova-Zadnikova et al. reduced frequency of serum-specific IgE allergies later in life (after 10 and 20 years) [45].

Gerasimov et al. conducted a study to assess the clinical efficacy and impact of Lctbs acidophilus DDS-1 and Bfdbm lactis UABLA-12 with fructooligosaccharide on peripheral blood lymphocyte subsets in preschool children with moderate-to-severe AD. In a randomized, double-blind, placebo-controlled, and prospective trial of 90 children aging 1–3 years with moderate-to-severe AD who were treated with a mixture of probiotics with fructooligosaccharide for 8 weeks versus placebo at the final visit, the percentage significant decrease in SCORAD was 33% in the probiotic group compared with 19% in the placebo group. Children receiving probiotics showed a greater decrease in the mean SCORAD score than did children from the placebo group at week 8. The administration of a probiotic mixture and fructooligosaccharide was associated with significant clinical improvement in children with AD, with corresponding lymphocyte subset changes in peripheral blood [46].

In brief, here, probiotics were more likely to be effective in treating moderately severe AD as well as mild atopic diseases. Although not every study result above was significant, the effect of probiotics did not seem to be greater just in the IgE-sensitized group than in the non-IgE-sensitized group. Nevertheless, there have been several reports in the literature showing no effect of probiotics, which are being discussed in the section below. 

#### 3.2.3. No Therapeutic or Preventative Effect of Probiotics in AD Regardless of IgE Sensitization

It is striking that the proportion of children with AD and allergic sensitization such as in the study of Taylor [49] and Huurre et al. [97] was significantly higher in the probiotic group. In Taylor et al.'s trial, probiotic supplementation postnatally failed to reduce the risk of AD and increased the risk of allergen sensitization in high-risk children. Newborns of women with allergy (*n* : 231) received either Lctbs acidophilus (LAVRI-A1) or placebo daily for the first 6 months of life. Children were assessed for AD and other symptoms at 6 and 12 months and had allergen skin prick tests at 12 months of age. At 6 and 12 months, AD rates were similar in the probiotic and placebo groups. At 12 months, the rate of sensitization was significantly higher in the probiotic group. The presence of culturable Lactobacilli or Bfdbm in stools in the first month of life was not associated with the risk of subsequent sensitization or disease; however, the presence of Lctbs at 6 months of age was associated with increased risk of subsequent cow's milk sensitization. Early probiotic supplementation with Lctbs acidophilus did not reduce the risk of AD in high-risk infants and was associated with increased allergen sensitization in infants receiving supplements. There were 3 major differences between Taylor's study and the others. The type of probiotic product (Lctbs acidophilus), the supplementation period (1 year), and the timing of the introduction of the probiotic were different. Taylor et al. administered the probiotic supplement postnatally, while other studies administered probiotics before and after birth. Prenatal supplementation may prove to be crucial for the preventative benefit of probiotics in this disorder. The data from Taylor et al.'s study point in the same direction regarding allergic sensitization, also suggesting that the use of probiotics for primary prevention must be exercised with caution [49].

Similarly, a randomized, double-blind, placebo-controlled, and prospective trial by Kopp et al. of probiotics for primary prevention did show no clinical effects of LGG supplementation; 105 pregnant women from families with ≥1 member (mother, father, or child) with an atopic disease were randomly assigned to receive either the probiotic LGG or placebo. The supplementation period started 4 to 6 weeks before expected delivery, followed by a postnatal period of 6 months. The primary endpoint was the occurrence of AD at the age of 2 years. Secondary outcomes were severity of AD, recurrent episodes of wheezing bronchitis, and allergic sensitization at the age of 2 years. Notably, children with recurrent (≥5) episodes of wheezing bronchitis were more frequent in the LGG group (26%), as compared with the placebo group (9%). As a result, supplementation with LGG during pregnancy and early infancy neither reduced the incidence of AD nor altered the severity of AD in affected children but was associated with an increased rate of recurrent episodes of wheezing bronchitis. No difference was observed between both groups in total IgE concentrations or numbers of specific sensitization to inhalant allergens [50].

Furthermore, prenatal probiotic LGG treatment during pregnancy was not associated with reduced risk of eczema or IgE-associated eczema in a RCT by Boyle et al. [47, 48]. In a recent study, 250 pregnant women were recruited carrying infants at high risk of allergic disease to a RCT of probiotic supplementation (LGG) from 36 weeks of gestation until delivery. Grüber et al.'s study also did not show any effect of LGG in infants with AD regardless of their IgE sensitization status [51].

However, a study from the Netherlands by Brouwer et al. and another study from Germany by Fölster-Holst et al. showed no effect of LGG in infants with AD regardless of their IgE sensitization status. In a study conducted by Brouwer et al., after 4–6 weeks of baseline and double-blind and placebo-controlled challenges for diagnosis of cow's milk allergy, infants less than 5 months old with AD received a hydrolyzed whey-based formula as placebo (*n* : 17) or were supplemented with either Lctbs rhamnosus (*n* : 17) or LGG (*n* : 16) for 3 months. No statistically significant effects of probiotic supplementation on SCORAD, sensitization, inflammatory parameters, or cytokine production between groups were found. No clinical or immunological effects of the probiotic bacteria used in infants with AD were found [52]. A similar prospective study by Fölster-Holst et al. was performed to reassess the efficacy of orally administered LGG in infants with AD. In a randomized, double-blind, and placebo-controlled study, 54 infants aging 1–55 months with moderate-to-severe AD were randomized to receive LGG or placebo during an 8-week intervention phase. At the end of treatment, there were no significant differences between the groups with respect to clinical symptoms (SCORAD, pruritus, and sleep loss), immunological parameters, or health-related quality of life of the parents [53]. Additionally, Soh et al. in a clinical trial involving 253 infants with a family history of allergic disease utilized probiotic supplementation (Bfdbm longum + Lctbs rhamnosus) in the first 6 months of life in Asian infants at risk and evaluated the effects on eczema and atopic sensitization at the age of 1 year. Early life administration of a cow's milk formula supplemented with probiotics showed no effect on prevention of eczema or allergen sensitization in the first year of life in Asian infants at risk of allergic diseases [54].

A randomized, double-blind, and placebo-controlled study was conducted in 34 adult-type AD subjects who were treated with conventional topical corticosteroid and tacrolimus. In these kinds of patients, heat-killed Lctbs paracasei K71 (LAB diet) may have been shown to have some benefits as a complementary therapy for adult AD patients who were managed with the conventional treatment [98].

In a double-blind, placebo-controlled, and crossover study, Bfdbm animalis subsp. lactis LKM512 yogurt was given for 4 weeks to 10 adult AD patients (4 males + 6 females; average age: 22 years) who were diagnosed with moderate AD. Scores of itching and burning tended to improve to a greater extent by LKM512 yogurt consumption than by placebo consumption. LKM512 yogurt consumption may be effective against intractable adult-type AD [99].

LGG was the mostly used probiotic species in these studies. Firstly used by Kalliomäki et al. [4] with a success, however, other groups including Brouwer, Boyle, Kopp et al., Grüber et al., and Fölster-Holst et al. [47, 50–53] could not demonstrate any benefit in AD. For instance, Kopp et al. have shown that the probiotic LGG has no preventative effect on the development or the severity of AD at the age of 2 years in a German population of infants at high risk. Instead, there was a significantly higher risk of ≥5 episodes with wheezing bronchitis during the first 2 years in the LGG group, as compared with placebo. There were several methodological differences between these studies: Kopp et al. adapted the protocol of Kalliomäki et al. and continued to supplement LGG for 3 months after birth to the breastfeeding mothers and the following 3 months only to the neonates. This modification was made to achieve a more consistent probiotic delivery. Second, Finnish mothers received supplementation during the last 4 weeks of pregnancy, whereas pregnant women in this population commenced with LGG or placebo for 4 to 6 weeks. They extended the prenatal supplementation period, because a 4-week period is thought to be possibly too short for the suspection of the in utero effects of LGG supplementation. Also, a population in the study by Kopp et al. was being of higher risk compared with the Finnish population, which might account for the differing results. And more infants with older siblings were recruited compared with the Finnish study. Lastly, the Finnish and German populations are of different genetic backgrounds. 

In summary, there is unsatisfactory but fairly promising evidence to recommend the addition of probiotics to foods for prevention and treatment of AD [100]. Nonetheless, there is a large amount of conflicting data on the preventative/therapeutic effects of probiotics in especially human clinical trials of AD. Results from these trials, meta-analyses, and systematic reviews that combine results of studies from different types of probiotics to examine the effects in any disease should be interpreted with caution. One may quickly recognize the degree of heterogeneity among the different probiotic studies as well. Very few studies were similar in design. For instance, several different probiotic strains with different dosing regimens were used [101]. And some probiotic studies suggest short-term statistically significant improvement in SCORAD scores and no sustained benefit from continued ingestion. Consequently, subgroup analysis became critical in understanding the outcomes of the studies. Not all individuals in clinical trials receiving the probiotic agent benefited, but subsets of these patients, mainly those with moderate disease activity and IgE-associated disease (atopic eczema), seemed to have benefited the most.

## 4. Conclusion

Currently, probiotics do not have a proven role in the prevention or therapy of allergic skin disorders. No single probiotic supplement or group of probiotic supplements has been yet demonstrated to efficiently affect the course of any allergic disease or manifestation. Therefore, probiotics cannot be recommended generally for primary prevention/therapy of allergic skin disorders [102]. If probiotics are used in patients with allergic skin disorders for any reasontherapy or prevention-cautionary approach ought to be taken. 

## Figures and Tables

**Table 1:** The various effects of different probiotic strains, referred to in this paper, on allergic skin conditions including atopic dermatitis, atopic dermatitis-like skin lesions, and allergic contact dermatitis in experimental (animal) studies are shown.

References	Probiotic species	Types of dermatitis in murine	Outcomes
		*Atopic dermatitis (AD) *	
Watanabe et al. [11]	Lctbs delbrueckii subsp. lactis	Atopic dermatitis	↓
Hayashi et al. [12]	Lactic acid bacteria	Atopic dermatitis	↓
Won et al. [13]	Lctbs plantarum	House-dust mite-induced AD	↓
Sawada et al. [14]	LGG	Atopic dermatitis	↓
Ogawa et al. [15]	Lctbs casei subsp. casei	Atopic dermatitis	↓
Marsella et al. [16, 17]	LGG	Atopic dermatitis	↓
		*AD-like lesions (trinitrochlorobenzene sensitization) *	
Viljanen et al. [18]	Lctbs acidophilus	Atopic dermatitis-like lesions	↓
Tanaka et al. [19, 20]	Lctbs rhamnosus	Atopic dermatitis-like lesions	↓
		*AD-like lesions (picrylchloride sensitization) *	
Ogawa et al. [15]	Lctbs casei subsp. casei	Atopic dermatitis-like lesions	↓
Wakabayashi et al. [21]	Lactic acid bacteria	Atopic dermatitis-like lesions	↓
Segawa et al. [22]	Lctbs brevis	Atopic dermatitis-like lesions	↓
		*Allergic contact dermatitis (dinitrofluorobenzene sensitization) *	
Park et al. [23]	Lctbs sakei probio-65	(1-Chloro-2,4-dinitrobenzene)-induced allergic dermatitis	↓
Chapat et al. [24]	Lctbs casei	Allergic contact dermatitis	↓
Hacini-Rachinel et al. [25]	Lctbs casei	Allergic contact dermatitis	↓
Weise et al. [26]	Escherichia coli Nissle 1917	Allergic contact dermatitis	↓

Lctbs: Lactobacillus; Bfdbm: bifidobacterium; LGG: Lactobacillus rhamnosus GG; ↓: decrease in symptoms or positive effect.

**Table 2:** The various effects of different probiotic strains, referred to in this paper, in (human) clinical allergic skin conditions such as atopic and nonatopic eczema are shown.

References	Probiotic species	Types of atopic dermatitis	Outcomes
		*Atopic (IgE-associated) Eczema *	
Majamaa and Isolauri [3]	LGG	Food-sensitized eczema	↓
Viljanen et al. [18]	LGG	Atopic eczema/dermatitis syndrome	↓
Rosenfeldt et al. [27]	Lctbs rhamnosus + Lctbs reuteri	Atopic eczema	↓
Sistek et al. [28]	Lctbs rhamnosus + Bfdbm lactis	Eczema, food-sensitized atopy	↓
Kukkonen et al. and Kuitunen et al. [29, 30]	Mix (LGG, Lctbs rhamnosus LC705, Bfdbm breve, and Propionibacterium)	Atopic eczema	↓
Kuitunen et al. [30]	Lctbs + Bfdbm + Propionibacteria	IgE-associated allergy	↓
Abrahamsson et al. [31]	Lctbs reuteri	Atopic eczema	↓
Isolauri et al. [32, 33]	Bfdbm or Lctbs	Food (cow's milk) allergy	↓
Wickens et al. [34]	Lctbs rhamnosus	IgE-associated eczema	↓
		*Nonatopic Eczema *	
Kalliomäki et al. [4]	LGG	Atopic dermatitis	↓
West et al. [35]	Lctbs casei F19	Atopic dermatitis	↓
Woo et al. [36]	Lctbs sakei	Atopic dermatitis	↓
Weston et al. [37]	Lctbs fermentum	Atopic dermatitis	↓
Hoang et al. [38]	Lctbs rhamnosus	Atopic dermatitis	↓
Hattori et al. [39]	Bfdbm breve	Atopic dermatitis	↓
Wickens et al. [34]	Lctbs rhamnosus, Bfdbm animalis (Bb-12)	Atopic dermatitis	↓
Marschan et al. [40]	Mix (LGG, Lctbs rhamnosus LC705, Bfdbm breve, and Propionibacterium)	Atopic dermatitis	↓
Niers et al. [41]	Bfdbm bifidum, Bfdbm lactis, and Lactococcus lactis	Atopic dermatitis	↓
Kim et al. [42]	Bfdbm bifidum, Bfdbm lactis, and Lctbs acidophilus	Atopic dermatitis	↓
Dotterud et al. [43]	LGG, Lctbs acidophilus, and Bfdbm animalis (Bb-12)	Atopic dermatitis	↓
Böttcher et al. [44]	Lctbs reuteri	Atopic dermatitis (sensitization)	↓
Lodinova-Zadnikova et al. [45]	Escherichia coli	Atopic dermatitis (IgE allergies)	↓
Gerasimov et al. [46]	Lctbs acidophilus and Bfdbm lactis	Atopic dermatitis	↓
		*Eczema (atopic dermatitis) *	
Boyle et al. [47, 48]	LGG	Atopic dermatitis	*↔*
Kuitunen et al. [30]	Lctbs + Bfdbm + Propionibacteria	Atopic dermatitis	*↔*
Taylor et al. [49]	LGG or Lctbs acidophilus	Atopic dermatitis	*↔*
Kopp et al. [50]	LGG	Atopic dermatitis	*↔*
Grüber et al. [51]	LGG	Atopic dermatitis	*↔*
Brouwer et al. [52]	Lctbs rhamnosus	Atopic dermatitis	*↔*
Fölster-Holst et al. [53]	LGG	Atopic dermatitis	*↔*
Soh et al. [54]	Bfdbm longum + Lctbcs rhamnosus	Eczema and atopic sensitization	*↔*

Bfdbm: Bifidobacterium; Lctbs: Lactobacillus; LGG: Lactobacillus rhamnosus GG; ↓: decrease in symptoms or positive effect,

*↔*: no change in symptoms or no effect.

## Abbreviations

AD: Atopic dermatitis
Lctbs: Lactobacillus
LGG: Lctbs rhamnosus GG
SCORAD: Severity scoring of atopic dermatitis
Ig: Immunoglobulin
LAB: Lactic acid bacteria
TLR: Toll-like receptor
Th1: T-helper 1
DC: Dendritic cell
Treg: T regulatory
TNCB: Trinitrochlorobenzene
La1: Lctbs johnsonii NCC533
LPR: Lctbs rhamnosus CGMCC 1.3724
AEDS: Atopic eczema/dermatitis syndrome
Bfdbm: Bifidobacterium
RCTs: Randomized (placebo-) controlled trials.
